The article "Detection of Radiolabeled Inflammatory Cell Macrophage Subpopulations in Chronic Respiratory Diseases: Results from Preliminary Analyses" was published in 2022. Journal: Biomed Res Int.

# Detection of Radiolabeled Inflammatory Cell Macrophage Subpopulations in Chronic Respiratory Diseases: Results from Preliminary Analyses

**DOI:** 10.1155/2022/9470845

**Published:** 2022-10-06

**Authors:** Abjal Pasha Shaik, Asma Sultana Shaik, Manal Abudawood, Achraf Al Faraj

**Affiliations:** ^1^Department of Clinical Laboratory Sciences, College of Applied Medical Sciences, King Saud University, Riyadh, Saudi Arabia; ^2^Prince Naif Health Research Center, College of Medicine, King Saud University, Riyadh, Saudi Arabia; ^3^Chair of Medical and Molecular Genetics Research, Department of Clinical Laboratory Sciences, College of Applied Medical Sciences, King Saud University, Riyadh, Saudi Arabia; ^4^College of Pharmacy, American University of Iraq - Baghdad (AUIB), Baghdad, Iraq

## Abstract

Chronic respiratory diseases (CRDs) like asthma and chronic obstructive pulmonary disease (COPD) are the leading causes of morbidity and mortality worldwide. Alveolar macrophages (AM) are immune cells that exist in different polarization states/phenotypes and have been shown to play a critical role during an inflammatory process. In this paper, differently polarized mouse bone marrow-derived macrophages (BMDM (M1-proinflammatory or M2-immunomodulator)) were radiolabeled with either 99mTc-D,L-hexamethylene-propyleneamine oxime (^99m^Tc-HMPAO), 2-deoxy-2-[18F] fluoro-D-glucose (^18^F-FDG), or ^67^Ga-citrate. Biocompatibility and *in vivo* biodistribution of radionuclide-labeled macrophages after intravenous injection were evaluated. Radioactivity measurements were performed using Packard Cobra Quantum 5002 Gamma Counter. Both M1 and M2 macrophages showed a higher uptake for ^18^F-FDG and ^99m^Tc-HMPAO, than ^67^Ga-citrate. M2 macrophages showed a higher uptake of radionuclides than M1 macrophages. The used radionuclides were biocompatible for both M1 and M2 macrophages. At 2-hour postinjection, ^18^F-FDG-labeled M1 and M2 macrophages were found significantly higher in the lung of inflammatory animals (12.54 ± 1.58% and 14.13 ± 1.03%, respectively) than in control mice. Labeling macrophages with either ^18^F-FDG or ^99m^Tc-HMPAO did not affect their biodistribution. The results from these initial experiments indicate that radionuclide-labeled macrophages may allow a higher sensitivity detection in nuclear imaging techniques such as PET and SPECT. Further confirmatory studies are needed to noninvasively image radiolabeled BMDM to understand their role in the inflammatory processes inherent to CRDs.

## 1. Introduction

Chronic respiratory diseases (CRDs) represent a substantial economic burden on global health [1]. They are the leading cause of morbidity and mortality worldwide [2]. One of the most important cells involved in the inflammatory processes in the lungs of patients with CRDs is the tissue macrophages [3], also called as the alveolar macrophages. These cells often undergo polarization to form two phenotypes, the M1 or M2 macrophages based on the inflammatory process [1]. Considerable efforts have been made in the last few years to better understand the heterogeneity of macrophages, their role in lung inflammation and tissue remodeling, and the molecular mechanisms that regulate macrophage polarization and plasticity under both *in vitro* and *in vivo* conditions [4–6]. It has been reported that the polarization states of alveolar macrophages can have distinct functions [4, 7]. M1 macrophages have a proinflammatory action and are activated by IFN-*γ* alone or in conjunction with bacterial lipopolysaccharides (LPS). M2 macrophages have immunomodulating role; are activated by IL-4, IL-13, immune complexes, IL-10, and/or glucocorticoids; and promote wound healing and angiogenesis [8]. Often M1 and M2 macrophages undergo plasticity based on the types of cytokines present in the extracellular environment [9]. Based on the type of inflammatory responses, a specific subpopulation of macrophages may predominate. It is therefore important to clarify which distinct macrophage population increases or decreases after an inflammatory process and to elucidate the infection-induced modulation of M1 and M2 macrophage phenotypes *in vivo*.

Tracing macrophage migration during their recruitment to the sites of inflammation also makes them ideal vehicles to deliver contrast agents or therapeutic interventions [10]. However, the impact of radionuclide labeling on the specific phenotype of bone marrow-derived macrophages (BMDM), toxicity, labeling efficiency, and *in vivo* biodistribution has never been assessed. Investigating the *in vivo* biodistribution of radionuclide-labeled macrophages is needed in order to allow a higher sensitivity detection using nuclear imaging techniques such as PET and SPECT and to offer the possibility of using a variety of clinically tested imaging agents [11, 12].

In the current study, we investigated the *in vivo* biodistribution of radionuclide-labeled macrophages after intravenous injection with the aim of elucidating the uptake of radionuclides and evaluating the biocompatibility of BMDM subsets.

## 2. Materials and Methods

### 2.1. Animals

Female BALB/c mice (20-25 g) were obtained from the university's main animal care center at the College of Pharmacy, King Saud University, Riyadh, Kingdom of Saudi Arabia. All experiments were performed in accordance with the national guidelines for the care of laboratory animals and were approved by the ethics committee of the College of Applied Medical Sciences (agreement number: CAMS05/3334).

### 2.2. Polarization of Macrophages

M1 and M2 polarized bone marrow-derived macrophages (BMDM) were obtained as previously described [13]. Briefly, the bone marrow cells were obtained from the tibiae and femora of donor BALB/c mice and were resuspended in Iscove's modified Dulbecco's medium (IMDM) (Life technologies, CA, USA) supplemented with 100 U/mL penicillin-streptomycin and 10% fetal bovine serum (Merck Millipore, MA, USA). The cells were then incubated at 37°C for 7 days in the presence of 10 ng/mL of macrophage clone stimulating factor (R&D systems, Abingdon, UK) to obtain adherent nonpolarized-M0 macrophages. Macrophage polarization was induced by incubating adherent M0 cells for 20 h at 37°C in IMDM supplemented with 1 ng/mL LPS (Santa Cruz Biotechnology, Inc., CA, USA) and 10 ng/mL IFN-*γ* (R&D systems, Abingdon, UK) to obtain M1-polarized cells or with 10 ng/mL IL-10 and 20 ng/mL IL-4 (R&D systems, Abingdon, UK) to obtain M2-polarized macrophages.

### 2.3. Radionuclide Labeling of Bone Marrow-Derived Macrophages

For radionuclide labeling, the cells were incubated in phosphate-buffered saline (PBS) with either 99mTc-D,L-hexamethylene-propyleneamine oxime (^99m^Tc-HMPAO), 2-deoxy-2-[18F] fluoro-D-glucose (^18^F-FDG), or ^67^Ga-citrate for 30 min at 37°C with radioactive labeling concentration of 1 million count per minute (cpm).

### 2.4. Biocompatibility Evaluation

Cell viability of radiolabeled M1 and M2 macrophages was evaluated by MTT Cell Growth Assay Kit (Merck Millipore, MA, USA) according to the manufacturer's instructions, and plates were read using the Multiskan Go Microplate Spectrophotometer (Thermo Scientific, NH, USA). Absorbance was measured with a test wavelength of 570 nm and a reference wavelength of 630 nm. The relative percentage of cell viability for each condition was calculated related to control one.

### 2.5. LPS-Induced Pulmonary Inflammatory Model

LPS from *E. coli* 0111:B4 (Santa Cruz Biotechnology, Inc., CA, USA) was administered intratracheally into the mice lungs (0.5 mg/Kg) using MicroSprayer® Aerosolizer (PennCentury, Pennsylvania, USA) to develop inflammation. At 48 hours after LPS challenge, bronchoalveolar lavage fluid was collected and centrifuged for 10 min at 300*g*, and the pellets resuspended in 1 mL PBS.

### 2.6. Biodistribution after Intravenous Injection

To assess the biodistribution of intravenously injected BMDM in control and inflammatory mice model, M1 and M2 macrophages were labeled with either ^99m^Tc-HMPAO or ^18^F-FDG radionuclides. The control and inflammatory mice models were intravenously injected with either M1 macrophages (labeled with either ^99m^Tc-HMPAO or ^18^F-FDG), M2 macrophages (labeled with either ^99m^Tc-HMPAO or ^18^F-FDG), or free radionuclides (^99m^Tc-HMPAO or ^18^F-FDG) as positive control (*n* = 3 for each group with a total of 36 mice).

At 2-hour postinjection, animals were dissected and organs of interest (i.e., lung, liver, spleen, and kidneys) were removed. Radioactivity measurements (percentage of injected dose [%ID] per gram) were then performed using Packard Cobra Quantum 5002 Gamma Counter equipped with a high-quality LCD display. The Cobra Quantum 5002 system also guarantees fast throughput with its fully automatic cassette-driven system and high detector efficiency. This Quantum 5002 Gamma Counter is designed with a single 2-inch Nal through-hole detector, a 2000 keV energy range, and a 750-sample capacity.

### 2.7. Statistical Analysis

Unless otherwise stated, data presented as the mean and standard deviation were analyzed by nonparametric statistical tests (SPSS, IL, USA): Kruskal-Wallis' test for unpaired groups and Friedman's test for comparison between different time points. A *p* value < 0.05 was considered significant for all tests.

## 3. Results

### 3.1. Quantification of Radionuclide Uptake by BMDM Subsets

Quantification of the uptake of radionuclides by either M1 or M2 macrophages revealed a higher uptake for ^18^F-FDG and ^99m^Tc-HMPAO, respectively, compared with ^67^Ga-citrate (Figure 1). M2 macrophages showed a higher uptake of the different radionuclides compared to M1 macrophages.

### 3.2. Biocompatibility Evaluation

All the used radionuclides, under the applied experimental conditions (i.e., labeling concentration and duration), were found to be biocompatible for both M1 and M2 macrophages with higher than 95% cell viability (Figure 2).

### 3.3. Biodistribution of Intravenously Injected Radionuclide-Labeled BMDM

Although the viability with the three radionuclides was >95%, the percentage of ^67^Ga-citrate uptake by M1 or M2 macrophages was much lower than either ^99m^Tc-HMPAO or ^18^F-FDG. Hence, we did not perform biodistribution analysis with ^67^Ga-citrate. Interestingly, at 2-hour postinjection, ^18^F-FDG-labeled M1 and M2 macrophages were significantly higher in the lungs of inflammatory mice (12.54 ± 1.58% and 14.13 ± 1.03%, respectively) compared to M1- and M2-labeled macrophages in the control mice and free injected FDG in the control and inflammatory mice (Figure 3). In addition, a higher dose of free FDG in both control and lung inflammation groups was detected in the spleen with no substantial variation observed in the liver and kidneys among groups (Figure 3). A same profile was observed with ^99m^Tc-HMPAO, which confirms that labeling macrophages with either ^18^F-FDG or ^99m^Tc-HMPAO did not affect their biodistribution.

## 4. Discussion

Alveolar macrophages are markedly increased in CRDs [14]. They have the ability to migrate to the inflammatory sites and deliver contrast agents for diagnosis or drugs as therapeutic modalities [13]. Therefore, the visualization of the migration of these cells using a noninvasive imaging modality to understand the physiological process in CRDs is required for both diagnostic purposes and for the evaluation of therapeutic interventions. Among the different strategies for imaging inflammatory processes, radionuclides labeling has been recognized as the most promising due to the potential for the early detection and diagnosis improvement.

Investigation of the *in vivo* biodistribution of radionuclide-labeled macrophages enables these cells to be used for ultrasensitive detection using nuclear imaging techniques to understand host associated with cell-mediated diagnosis and therapy. To assess the *in vivo* biodistribution of macrophages in an inflammatory lung model with a high sensitivity detection, the uptake of different PET or SPECT radionuclides by BMDM subpopulations was quantified in a preliminary investigation. In addition, the biocompatibility of radiolabeled macrophages was evaluated. Labeling M1 or M2 macrophages with either ^18^F-FDG (PET radionuclide) or ^99m^Tc-HMPAO (SPECT radionuclide), chosen based on preliminary evaluations (data not shown), revealed a high uptake while maintaining the viability and proliferation profile of radiolabeled macrophages. A high uptake was detected with M2 macrophages compared to M1 subpopulation consisting their higher phagocytic capacity in line with their role as debris scavengers.

After their intravenous injection, ^18^F-FDG- or ^99m^Tc-HMPAO-labeled M1 and M2 macrophages were found to preferentially home to the inflammatory sites in the lungs of inflammatory mice with a higher radioactivity measured in the lungs of LPS induced groups at 2-hour postinjection. These observations confirmed that labeling cells using ^18^F-FDG and ^99m^Tc-HMPAO radionuclides, under the used experimental conditions, did not affect the biodistribution of macrophage subpopulations. This preliminary imaging study provided evidence of the biodistribution of macrophages in organs after their excision from mice. *In vivo* biodistribution metabolic studies in living animals can provide confirmation on the potential mechanisms and the underlying pathways associated with the biodistribution of radiolabeled macrophages in inflammatory process along with an understanding of the potential use of nuclear medicine noninvasive imaging in CRDs like asthma and COPD. Further studies using noninvasive imaging of radiolabeled macrophages using PET and SPECT will confirm the radioactivity measurements in the different organs and asses the ultrasensitivity of nuclear imaging modalities in the detection of injected macrophages into the inflammatory sites.

## 5. Conclusions

This novel study showed that ^18^F-FDG and ^99m^Tc-HMPAO radionuclides could be used for identifying the biodistribution of macrophages in the lung inflammatory sites. This can have immense scientific potential as the use of radiolabeled macrophages could provide a noninvasive imaging method with both diagnostic and therapeutic implications for CRDs.

## Figures and Tables

**Figure 1:** Percentage of ^99m^Tc-HMPAO, ^18^F-FDG, or ^67^Ga-citrate uptake by M1 or M2 macrophages. Error bars are standard deviation of triplicates.

**Figure 2:** Percentage of viability (assessed by MTT) of M1- and M2-labeled macrophages with either ^99m^Tc-HMPAO, ^18^F-FDG, or ^67^Ga-citrate radionuclides. Error bars are standard deviation of triplicates.

**Figure 3:** Biodistribution of ^18^F-FDG-labeled M1 and M2 macrophages compared to free injected ^18^F-FDG in the control and inflammatory mice model having received intrapulmonary LPS exposure.

## Data Availability

The data will be given by the authors on request.
